# The impact of insecticides and plant extracts on the suppression of insect vector (*Bemisia tabaci*) of Mungbean yellow mosaic virus (MYMV)

This article has been retracted.

**DOI:** 10.1371/journal.pone.0256449

**Published:** 2021-09-16

**Authors:** Muhammad Younas, Huasong Zou, Tasmia Laraib, Nasir Ahmad Rajpoot, Nasir Ahmad Khan, Anas Ahmad Zaidi, Ghalib Ayaz Kachelo, Muhammad Waqar Akhtar, Shoukat Hayat, Abdullah M. Al-Sadi, Samy Sayed, Hosny Kesba, Mohammad Javed Ansari, Ali Tan Kee Zuan, Yunzhou Li, Muhammad Arif

**Affiliations:** 1 Department of Plant Pathology, University of Agriculture Faisalabad, Faisalabad, Pakistan; 2 College of Plant Protection, Fujian Agriculture and Forestry University, Fuzhou, China; 3 Institute of Molecular Biology and Biotechnology, The University of Lahore, Lahore, Pakistan; 4 Department of Plant Pathology, The Islamia University of Bahawalpur, Bahawalpur, Pakistan; 5 Department of Soil Science, The Islamia University of Bahawalpur, Bahawalpur, Pakistan; 6 Department of Forestry, The Islamia University of Bahawalpur, Bahawalpur, Pakistan; 7 Department of Plant Sciences, College of Agricultural and Marine Sciences, Sultan Qaboos University, Alkhoud, Oman; 8 Department of Science and Technology, University College-Ranyah, Taif University, Taif, Saudi Arabia; 9 Zoology and Agricultural Nematology Department, Faculty of Agriculture, Cairo University, Giza, Egypt; 10 Department of Botany, Hindu College Moradabad (Mahatma Jyotiba Phule Rohilkhand University Bareilly), Moradabad, India; 11 Department of Land Management, Faculty of Agriculture, Universiti Putra Malaysia, UPM, Selangor, Malaysia; 12 Department of Plant Pathology, College of Agriculture, Guizhou University, Guiyang, Guizhou, China; 13 Department of Plant Protection, Fujian Agriculture and Forestry University, Fuzhou, China; Ghazi University Dera Ghazi Khan, PAKISTAN

## Abstract

Mungbean yellow mosaic virus (MYMV) is an important constraint in successful production of mungbean (*Vigna radiata* L.) in many countries, including Pakistan. The MYMV spreads by insect vector whitefly (*Bemisia tabaci* Gennadius). The use of resistant cultivars is the most effective management tactics for MYMV. Twenty mungbean varieties/lines were screened against insect vector of MYMV under field condition in the current study. Resistance levels for varieties/lines were assessed through visual scoring of typical disease symptoms. Furthermore, the impacts of two insecticides ‘Imidacloprid’ and ‘Thiamethoxam’ and two plant extracts, i.e., neem (*Azadirachta indica*), and Eucalyptus (*Eucalyptus camaldulensis*) were tested on the suppression of whitefly. Field screening indicated that none of the tested varieties/lines proved immune/highly resistant, while significant variations were recorded among varieties/lines for resistance level. All varieties/lines were systemically infected with MYMV. The varieties ‘AARI-2006’ and ‘Mung-14043’ were considered as resistant to MYMV based on visual symptoms and the lowest vector population. These varieties were followed by ‘NM-2006’ and ‘NL-31’, which proved as moderately resistant to MYMV. All remaining varieties/lines were grouped as moderately to highly susceptible to MYMV based on visual symptoms’ scoring. These results revealed that existing mungbean germplasm do not possess high resistance level MYMV. However, the lines showing higher resistance in the current study must be exploited in breeding programs for the development of resistant mungbean varieties/lines against MYMV. Imidacloprid proved as the most effective insecticide at all concentrations to manage whitefly population. Therefore, use of the varieties with higher resistance level and spraying Imidacloprid could lower the incidence of MYMV.

## Introduction

Mungbean (*Vigna radiata* L.), a member of the Fabaceae is an important source of vitamins, carbohydrates and protein for human globally [1–4]. It is commonly known as mash bean, green bean, green gram and golden gram [5]. Mungbean is an ancient, conventional and the cheapest pulse fulfilling protein demands of developing countries. It originates in Asia and was firstly introduced in south China during the early 18^th^ century. It is widely cultivated in Pakistan, Philippine, India, Burma and Thailand from previous three decades [6]. Later on, it has been introduced to West Indies, the US, and East and Central Africa [7]. Mungbean is considered as the second most important pulse crop after chickpea in Pakistan; however, its average yield in the country is low compared to other countries in the world. Several factors such as low yielding cultivars, traditional methods of cultivation, lack of irrigation facilities and particularly outbreaks of numerous diseases are responsible for low mungbean yield in the country [8, 9].

Numerous viral, bacterial and fungal diseases infest mungbean [10] and viral diseases are a potential threat to its successful production. Mungbean yellow mosaic virus (MYMV) is serious diseases of mungbean widely observed in Pakistan, India, Bangladesh Philippines, Thailand and Sri Lanka [5, 11–13]. The incidence of MYMV varies from 4–40% and reaches 100% depending on location and crop variety in Pakistan [14, 15]. The MYMV belongs to family *Geminiviridae* and genus *Begomovirus*. It was firstly identified in 1955 and noticed that whitefly (*Bemisia tabaci*) is responsible for the transmission of MYMV. This virus cannot be transmitted through seed, sap or mechanically. However, Thailand strain of this virus is capable of mechanical transmission [16, 17].

Appearance of small, irregular yellow spots are the typical symptoms of MYMV. These lesions get enlarged and lead to complete yellowing of leaves at later growth stages of crop. The growth of infected plants become stunted resulting in the production of few flowers. Disease severity mainly depends on successful infection and may reach 85% [18, 19].

Different management strategies are opted by farmers and researchers to manage MYMV. However, use of resistant varieties is the most economical and environment-friendly management option for MYMV [4, 14, 20, 21]. Management of whitefly through chemicals (pesticides, insecticides) can significantly reduce disease incidence. According to integrated pest management (IPM) strategy, chemicals should be applied after the appearance of first disease symptom on host [22, 23] for high yield and quality. However, use of insecticides results in the evolution of insecticides’ resistant insect populations and exerts negative effects on environment. Therefore, alternative management methods have gained increased importance in the recent decades. The use of plant extracts have given promising results in the management of various insect species.

The use of resistance cultivars necessitates their identification first under field conditions. Unfortunately, resistance level of recently developed mungbean varieties and lines against MYMV is unknown. Furthermore, lowering the vector population could help in lowering the disease incidence. Therefore, major objective of the current study determine the resistance level of available mungbean varieties/lines against MYMV under field conditions. Finding the relationship between the population of insect vector and MYMV was the second objective. Testing the impacts of different insecticides on vector and subsequent MYMV suppression was the last objective. It was hypothesized that the varieties/lines will significantly differ in their resistance level to MYMV. Furthermore, the plant extracts will effectively suppress whitefly population and MYMV incidence comparable to insecticides. The results will help to select the suitable varieties/lines for resistance improvement and selection of environment-friendly management option for whitefly in mungbean.

## Materials and methods

### Collection of varieties/lines and sowing

Mungbean germplasm was collected from Ayub Agriculture Research Institute (AARI), Faisalabad, Pakistan. Field screening and efficacy experiments were conducted at the experimental area of Department of Plant Pathology, University of Agriculture Faisalabad, Pakistan during 2018. Sixteen mungbean lines, i.e., (‘TM 1428’, ‘NI 31’, ‘M 303’, ‘M 1977’, ‘E 39’, ‘E 182/2’, ‘E 86’, ‘RA 8K’, ‘LNO 54’, ‘LNO 127’, ‘LNO 37’, ‘LNO 11’, ‘M 97001’, ‘M 632’, ‘M 002’ and ‘A 6601’) were used in the study. Seeds were manually sown by keeping plant-to-plant distance of 15 cm and row-to-row distance of 30 cm. One line of susceptible check variety was cultivated as spreader after every third row of tested lines/varieties. The experiment was conducted according to randomized complete block design (RCBD) with three replications.

### Preparation and application of insecticides and plant extracts

The main objective of the study was to evaluate different insecticides and plant extracts on whitefly population and subsequently incidence of MYMV. The insecticides were purchased from Syngenta Pakistan Pvt. Ltd. and plant extracts were prepared in the laboratory. The plant extracts were prepared by following the method of Venkatesan et al. [24]. The mature leaves (1000 g each) neem (*Azadirachta indica*) and Eucalyptus (*Eucalyptus camaldulensis*) were homogenized independently in pre-chilled mortar and pestle and through applying chilled sterilized distilled water. Both extracts were filtered through four layer of moistened muslin cloth. The final volume of the extracts was adjusted to 1:1 with the help of distilled water. The whole filtrate was centrifuged at 15000 × g at 48°C for 15 minutes. The obtained supernatant was designated as concentrated botanical extract of both species. Serial dilutions to make the volume of 1:10 were completed for both extracts as this concentration is recommended for most of the studies. Additionally, we added two reduced concentrations of the extracts, i.e., half of the recommended and one third of the recommended to assess whether lower dose are suitable for suppressing the population of whitefly. Two insecticides, i.e., (‘Thiamethoxam’ and ‘Imidacloprid’) were applied at three different concentrations, i.e., (recommended, half of the recommended and one third of the recommended) to test their impacts on whitefly population and subsequently MYMV infestation. The data relating to MYMV incidence and whitefly population was recorded by visually assessing the plants and counting the number of whitefly individuals, respectively. Disease incidence was evaluated by following the standard disease rating scale [25, 26]. Response of different mungbean lines was determined based on percent disease infestation and lines were scored by using recommended 0–5 arbitrary scale (Table 1) at reproductive stage [27–29].

**Table 1:** Disease rating scale used for the determination of MYMV infestation on tested mungbean lines/varieties.

Disease score/rating	Infestation (%)	Resistance level	Response group
0	Plants free from disease	Immune/highly-resistant	I/HR
1	1–10%	Resistant	R
2	11–20%	Moderately-resistant	MR
3	21–30%	Moderately-susceptible	MS
4	30–50%	Susceptible	S
5	Up to 50%	Highly-susceptible	HS

### Statistical analysis

The collected data were statistically analyzed by using SAS statistical software (SAS Institute, 2008). The data were analyzed by one-way analysis of variance (ANOVA). The normality in the data was tested first, which indicated a non-normal distribution. Therefore, data were transformed by Arcsine transformation technique. Means were separated by least significant difference (LSD) test at 5% probability level where ANOVA indicated significant differences [30]. The data for the concentrations of extracts and insecticides were analyzed for each concentration, separately since these were not considered as a factor. Minimal dataset of the study is given in S1 Dataset.

## Results

### Response of mungbean varieties/lines to MYMV

None of the tested twenty varieties/lines proved highly-resistant/immune MYMV and whitefly. Two varieties/lines, i.e., ‘AARI-2006’ and ‘Mung-14043’ proved resistant, whereas ‘NM-2006’ and ‘NL-31’ were scaled as moderately-resistant. The lines ‘TM-1428’ and ‘M-6’ were moderately susceptible to MYMV. Seven out of twenty varieties/lines, i.e., ‘E-86’, ‘E-39’, ‘M-1977’, ‘8A-8k’, ‘LNO-154’, ‘LNO-11’ and ‘M-303’ proved susceptible to MYMV. The remaining seven varieties/lines, i.e., ‘E-182’, ‘M-97001’, ‘M-632-72’, ‘M-002’, ‘LNO-127’, ‘M-6601A’ and ‘LNO-37’ proved highly susceptible to MYMV during the current study (Table 2).

**Table 2:** Resistance level/response of mungbean varieties/lines according to the infection categories of MYMV disease rating scale.

Infection category	Disease rating	Number of varieties/lines	Varieties/lines
Highly resistant (HR)	0	0	0
Resistant (R)	1	2	‘AARI-2006’, ‘Mung-14043’
Moderately resistant (MR)	2	2	‘NM-2006’, ‘NL-31’
Moderately susceptible (MS)	3	2	‘TM-1428’, ‘M-6’
Susceptible (S)	4	7	‘E-86’, ‘E-39’, ‘M-1977’, ‘8A-8k’, ‘LNO-154’, ‘LNO-11’, ‘M-303’
Highly susceptible (HS)	5	7	‘E-182’, ‘M-97001’, ‘M-632-72’, ‘M-002’, ‘LNO-127’, ‘M-6601A’, ‘LNO-37’

### Response of mungbean varieties/lines to whitefly infestation

Two varieties/lines, i.e., ‘Mung-14043’ and ‘AARI-2006’ recorded the lowest whitefly population and expressed resistant response to MYMV followed by ‘NM-2006’ and ‘NL-31’, which were ranked as moderately-resistant to MYMV. The population density of whitefly on mungbean varieties/lines named ‘TM-1428’, ‘M-6’, ‘E-86’, ‘M-1977’, ‘LNO-54’, ‘M-303’, ‘LNO-11’ and ‘E-39’ ranged between 1–2.66 adults per plant. Similarly, the lines ‘M-97001’, ‘M-6601’, ‘E-182, M-8A’, ‘M-632’, ‘M-002’, ‘LNO-127’ and ‘LNO-37’ observed higher density of whitefly compared to the rest of the varieties/lines included in the study. The whitefly population density on these varieties, lines ranged between 3.33 and 5.00 adults per plant (Table 3).

**Table 3:** The population density of whitefly on different mungbean varieties/lines included in the study.

Varieties/lines	White fly population (adults plant^-1^)
‘TM-1428’	1.00
‘NL-31’	0.66
‘M-303’	2.33
‘M-1977’	1.66
‘E-39’	2.66
‘E-182’	3.33
‘E-86’	1.33
‘8A-8k’	3.33
‘LNO-154’	1.66
‘LNO-11’	2.33
‘M-97001’	3.33
‘M-632-72’	4.00
‘M-002’	4.00
‘LNO-127’	4.33
‘M-6601A’	3.33
‘LNO-37’	5.00
‘AARI-2006’	0.33
‘NM-2006’	0.66
‘M-6’	1.00
Mung-14043	0.33
LSD_(0.05)_	1.98

### Effects of recommended doses of insecticides and plant extracts on MYMV infestation

Recommended doses of tested pesticides and plant extracts significantly lowered MYMV incidence as compared to control treatment. Mean number of infested plants by MYMV was the lowest for Imidacloprid (11.16%) followed by Thiamethoxam (20.16%), neem (20.16%) and *Eucalyptus* (30.08%). The highest number of infested plants by MYMV was recorded in control treatment. The mean disease incidence was lowest with the application of Imidacloprid insecticide compared to the rest of the treatments (Table 4).

**Table 4:** The impact of recommended doses of different insecticides and plant extracts on the incidence of MYMV.

Treatments	Disease incidence (%)
Imidacloprid	11.16 e
Thiamethoxam	20.16 d
Neem	23.91 c
Eucalyptus	30.08 b
Absolute Control	89.50 a
LSD 0.05	0.94

### Impact of different doses of insecticides and plant extracts on MYMV infestation

Different doses of insecticides and plant extracts significantly lowered the incidence of MYMV; however, the highest suppression was noted with the recommended doses. The disease incidence was increased with decreasing doses of all insecticides and plant extracts (Table 5). The lowest disease incidence was recorded for the recommended dose of Imidacloprid, whereas other two doses also exhibited the highest suppression compared to the respective doses of other insecticide and plant extracts. The control treatment observed the highest disease incidence (Table 5).

**Table 5:** The impact of doses of various insecticides and plant extracts on the incidence of MYMV under field conditions.

Disease incidence (%)			
Treatments	Recommended dose	Half of the recommended doses	One third of recommended dose
Imidacloprid	11.33 e	32.83 e	21.20 e
Thiamethoxam	22.33 d	45.05 d	30.91 d
Neem	24.93 c	48.00 c	35.16 c
Eucalyptus	28.75 b	53.16 b	38.58 b
Control	89.00 a	85.00 a	88.00 a
LSD 0.05	1.27	1.34	1.65

## Discussion

Viral diseases, including mungbean yellow mosaic virus (MYMV) drastically reduce yield of various legume crops. Screening of mungbean varieties/lines for MYMV-tolerance under field conditions confers the susceptibility of available lines to MYMV. The widespread susceptibility might be linked with the presence of disease vector (*Bemisia tabaci*) and favorable environmental conditions for disease development. The frequency of housefly outbreaks has been increased due to the development of insecticides resistance, which demands cultivation of resistant lines/varieties [31–33]. Identification of MYMV-resistant mungbean lines is an economic, environmental compatible and effective control strategy to combat MYMV [4, 34, 35].

The present study evaluated 20 mungbean lines/varieties against MYMV and their vector under field conditions. Field assessment revealed diverse resistance responses of the tested lines/varieties. All of the tested lines/varieties were infested by MYMV disease and whitefly. Results revealed that none of the tested variety/line was highly-resistant to MYMV. All the symptomatic plants were tested positive for MYMV compared to symptomless plants, which were tested negative. Significant differences in whitefly density were recorded among tested lines/varieties; however, none of the variety/line was completely free from whitefly population. Results indicated that ‘AARI-2006’ and ‘Mung-14043’ had resistant response to MYMV with minimum housefly population followed by ‘NM-2006’ and ‘NL-31’, which were moderately-resistant to MYMV. The remaining lines proved recorded moderately to highly-susceptible against MYMV.

It has been reported from previous studies that presence of MYMV resistance is rare in mungbean varieties/germplasm [33, 36–39]. Earlier studies have also reported that there is no immune/highly-resistant line to MYMV among the tested 247 lines [13, 16, 40]. Similarly, nine resistant lines were identified under field conditions among 83 tested lines against MYMV; however, none of them was categorized as highly-resistant [34, 41]. It is reported that two recessive genes control the mechanism of disease resistance in mungbean crop, while susceptibility is only controlled by a single recessive gene [26, 42]. It is clear that susceptibility is mainly dominant on resistance. Disease infestation was significantly increased by increasing vector population. Results of present study also revealed that low densities of whitefly can efficiently transmit begomoviruses [43, 44]. Disease infestation mainly depends on environmental condition, vector host presence, age of plant, host resistance to vector, soil condition, and inoculum level [45–48].

Identification of resistance source is useful for the selection of germplasm and exploit it in breeding programs for the development of resistant varieties/lines [49–51]. The use of resistant varieties/lines is regarded as the most appropriate way to manage MYMV. However, if disease appears suddenly in epidemic form then the farmers are bound and forced to use chemicals, which are quick in action against MYMV. Nonetheless, inappropriate use of chemicals cause health hazardous and various environmental issues. Therefore, insecticides and plant extracts were compared for their efficacy in suppressing whitefly and subsequently MYMV infestation. Imidacloprid proved more toxic to whitefly as compared to remaining insecticide and plant extracts and recorded minimum infestation to control. These results are in agreement with those who studied whitefly management [52–54]. Results of present study are supported by the work of [55, 56] who managed whitefly by using Imidacloprid. The current study also suggested that plant extracts are capable of suppressing whitefly and incidence of MYMV. Therefore, these can be combined with insecticide to lower the dose of the insecticide and subsequently decrease environmental and ecological impacts.

## Conclusion

This study concludes that none of the newly developed lines was highly resistant to MYMV; however, some of these were resistant. The resistant lines/varieties should be cultivated after their adaptability in various agro-ecological zones of the country. The highest suppression of whitefly population and incidence of MYMV was noted with the use of Imidacloprid insecticide. Nonetheless, neem extract were also effective in reducing whitefly population and MYMV. Therefore, impacts of Imidacloprid and neem extract combination must be evaluated in the future studies. The proper and timely application of new chemistry insecticides with combination of neem extracts could be viable approach to manage MYMV. However, this inference needs thorough testing before generalization.

## Supporting information

S1 Dataset Minimal dataset used to compute means and build tables presented in the current study. (XLSX)
